# Logistics Finance Collaborative Development Model Based on Machine Learning

**DOI:** 10.1155/2022/1591371

**Published:** 2022-09-24

**Authors:** Yuqin Wang

**Affiliations:** Department of Logistics Management, Xi'an International University, Xi'an 710077, China

## Abstract

In the context of rapid social development, a logistics financial model that can meet the financing needs of small and medium-sized enterprises and has high returns is widely used in all aspects of the logistics financial industry. Logistics finance is a new financing model that can effectively integrate logistics enterprises, financial companies, and financing institutions to achieve mutual benefit and win-win results. The uncertainty of financial information, the motivation of each business service object to pursue high returns in a short period of time, and the inadequate risk preuniversal conditions have led to credit risks in the development of logistics financial services. Promoting the close integration of improved neural network algorithms based on machine learning and logistics financial financing models is inseparable from the active cooperation of all aspects, the trust of various business service objects, and the construction of logistics financial information platforms. Based on machine learning, this paper analyzes and models the collaborative development of logistics finance, analyzes the original data, and constructs sample characteristics. Due to the small amount of information in part of the sample features, this causes problems such as overfitting in the process of model building. Therefore, we designed a new feature selection based on Pearson correlation coefficient and PCA. *Method*. Using this algorithm for feature selection, an integrated learning method is proposed. In order to solve the shortcomings of traditional neural network logistics algorithms, a neural network-based noncomplete vehicle path optimization mining model is proposed. By weighting the time domain length and spatial probability of logistics finance, the stable state of the neural network is restricted. Simulation results show that this method can effectively improve logistics efficiency and maximize the economic value of the transportation process.

## 1. Introduction

The logistics industry is a productive service-oriented industry. It is closely related to the stable operation of the real economy and has a strong correlation with the three major industries [1]. The services of the logistics industry can be said to be all-encompassing, almost including the circular flow of materials, semifinished products, and other resources in each link of the circular supply system such as purchase, manufacturing, and wholesale [2]. The refinement and perfection of the logistics industry has reduced the transportation threshold of the logistics industry and saved a lot of costs, so that many small- and medium-sized enterprises can choose suitable logistics services according to their actual situation, and the corresponding logistics finance has gradually developed. From the perspective of the applicants of logistics finance—small- and medium-sized enterprises, the existing resources can be integrated as a guarantee, and through the mobilization of logistics enterprises, use movable property resources to apply for loans from banks or other financial institutions. In this way, small- and medium-sized enterprises can obtain the funds needed for business operations [3]. Second, with the assistance and cooperation of logistics enterprises, banks or financial institutions can reduce the credit risk of logistics finance and obtain part of the benefits at the same time [4]. Finally, logistics companies can rely on comprehensive services to obtain profits. In addition, through China's partnership with financial companies and financing departments, it can help logistics companies to more deeply integrate into the production and supply system established by customers and enterprises [5]. At present, the modern logistics industry has contributed more and more to China's economic growth and has gradually become a pillar industry in the economic structure [6]. The optimization and adjustment of the logistics system structure is conducive to the rational allocation of regional resources. The rapid development of the logistics industry can not only stimulate the rapid growth of the Chinese economy, inject fresh blood into the Chinese market, but also promote employment of laborers [7].

## 2. Related Works

Previous research found through continuous research and investigation that as the banking industry's entry barriers continue to decrease, competition in the financial market has greatly intensified, which prompts banks and other financial institutions to consolidate their positions by continuously expanding their businesses [8]. However, due to the difficulty of managing and controlling credit risks for SMEs, they are still cautious in financing business. In China, the threshold for starting a logistics company is low, which has resulted in a large number of logistics companies in China, especially small logistics companies founded by individuals [9]. Under the background of this low-level competition, China's domestic logistics companies have low overall profit margins. In order to cope with this situation, logistics companies have to develop new value-added logistics services to expand profit margins and seek further development [10]. The literature believes that logistics finance is produced with the continuous development of the logistics industry, and it is an industrial integration with the highest degree of integration [11]. It aims at the efficient operation of capital flow and ensures the real-time update and sharing of information through effective management and control of the actual logistics situation. At the same time, a variety of financial products are used efficiently and reasonably to realize the flow and distribution of funds. The flow of funds is reflected in the entire logistics process, including deposits and loans, investment, trust leasing, insurance, securities issuance and trading, and logistics related to various intermediate businesses, which can be managed by banks and other financial institutions [12]. The literature pointed out that at present, various countries and regions in the world have various methods for establishing industry logistics demand forecasting models [13]. Each researcher has his own different ideas. They put forward their own opinions by analyzing the research objects and combining their own thinking. The core point of the literature is that the forecasting models established by most researchers are single and do not fully consider all the influencing factors related to logistics demand, which leads to unsatisfactory results from the forecasting model [14].

## 3. Machine Learning and Improved Neural Network Algorithm

### 3.1. Machine Learning Algorithm

Since its establishment in 1959, the vehicle scheduling problem has gradually become the focus of research and discussion in the field of combination optimization and operations research. So far, domestic and foreign researches in this field are mainly divided into three aspects: problem abstract modeling, basic problem decomposition, and algorithm solving. After years of research, the basic principles of various models and algorithms have become more and more perfect.

In the transportation logistics transportation process of the current class of problems-receiving point location is scattered, if blindly to transport, easy to cause waste of time cost, and transportation cost, so we need scientific distribution vehicle and route, through to the order information integration and road information research, make vehicle as convenient as possible after a series of receiving points, so as to achieve the shortest distance, the most saving time, the lowest fuel consumption cost, this way is called vehicle scheduling optimization. The main factors of this problem include distribution vehicle, distribution center, user demand, user location, constraint conditions, and objective function. The distribution center has K distribution vehicles of the same type, each with a capacity of *Q*, and there are a total of *N* customers, and *X* represents the corresponding demand of each customer. Vehicle scheduling needs to formulate a reasonable driving route, and the total cost is minimal, including time cost, distance cost, and transportation cost. Then, the basic mathematical model of vehicle scheduling optimization problem can be described as:

(1) $$\begin{array}{c} \min\;z=\underset{i}{\sum }\underset{j}{\sum }\underset{k}{\sum }c_{ij}*X_{ijk}\text{,}\\ X_{ijk}=\left\{\begin{array}{cc} 1 & vehicle\;k\;from\;DCi\;to\;j\\ 0 & other \end{array}\right.\text{,}\\ X_{ijk}=\left\{\begin{array}{cc} 1 & cehicle\;k\;serve\;i\\ 0 & other \end{array}\right.\text{,}\\ \underset{i}{\sum }qi*Y_{iK}\leq Q\;k=1,2,\ldots ,k\text{,}\\ \underset{j}{\sum }X_{ijk}=Y_{iK\;}i=1,2,\ldots \text{,}N\text{,}\\ \underset{i}{\sum }Y_{ik}=1,i=1,2\ldots N\text{,}\\ \underset{j}{\sum }X_{ijk}=Y_{jk}\;i=1,2,\ldots \text{,}N\text{.} \end{array}$$

The data used in the training in this article come from the Tmall e-commerce platform. The data are randomly selected user product interaction records from November 18, 2014, to December 18, 2014. In this article, the commodity purchase problem is a binary classification problem. By constructing certain characteristics of the sample, it can be determined whether the sample is a positive sample or a negative sample. A positive sample indicates that the user has purchased a product, and a negative sample indicates that the user has not purchased the product. In other words, we can determine whether to purchase the product through the relevant characteristics of the user.

In the predictive model, there is not much correlation with other data, so these data are features that are not used in the construction. The user's operation data and other data are not lost at a specific time. We consider using these raw data to build a machine learning sample data set.

In the research process of this article, the original data are only the user's operating data on the operating platform, and the number of feature values cannot be used as training samples in the machine learning process. In this case, we need to perform special processing on the original sample to convert it into useable sample data and extract sample features with higher utility value from it. Feature engineering is mainly divided into three parts: data processing, feature transformation, and feature selection. Data processing is mainly to convert raw data into machine learning training samples; feature transformation is to analyze the raw data of training samples to obtain high-dimensional and high-value features. Feature selection, as the name implies, is actually to screen all sample information, retain key information in high-dimensional samples, and delete those features that are less relevant and less informative, which greatly simplifies the fitting process. The three parts of feature engineering greatly reduce the difficulty of the data fitting process, not only fully and fully extract the core content of the sample but also improve the accuracy of the prediction model.

After the selection of data set is clarified, the characteristics of user operation data are extracted. For example, the amount of attention a user pays to a particular product over a period of time, including browsing and adding to the cart, the last time a user purchased that product, and the time between browsing and paying for a purchase. This data can then be used for machine learning.

Because there may be collinear relationship structural features and characteristics, which makes the model easy to fall into an overfitting state, we should try our best to eliminate features with a high degree of linear correlation and retain features with a large amount of information. Finally, we can get the Pearson correlation coefficient: capability. Usually, we need to determine the effect of the model, so we must use some methods to evaluate the rationality of the model. The following are two methods of machine learning model verification.

#### 3.1.1. Reserve Method

In this method, the data set *D* is proportionally divided into two mutually exclusive data sets, *S* represents the training set, and *T* represents the test set. The model is fitted through the training set *S*, and the test set *T* is used to generalize the error estimation. However, if the training set *S* occupies a large proportion, the obtained training model is close to the training model of the data set *D*, which leads to insufficient accuracy of the evaluation error of the test set. On the contrary, if the proportion of the test set *T* in the total data set *D* is much higher than the proportion of *S*, then it means that there is a large gap between the samples in the training set *D* and the samples in *T*. This leads to the training model not meeting the requirements of the original data model, which leads to a decrease in the accuracy of the evaluation error.

#### 3.1.2. Cross-Validation Method

The core idea of the “cross-validation method” is to divide a total data set *D* into *n* similar irrelevant subsets. Then choose one of the *n* subsets as the test set, and the remaining *n* − 1 subsets as the training set, and train the training set. This is done *n* times, the results obtained from these *n* times are averaged, and the final result is finally obtained. The process is shown in Figure 1.

We should pay special attention to the scope of the cross-validation method. This method is only suitable for the case of small data volume, but this method is not applicable when the computing power is low and the data volume is large.

### 3.2. Improved Neural Network Algorithm

The core of BP neural network learning is the reverse transmission of error information. The error estimation of each layer of BP neural network can be obtained by transmitting the error information layer by layer. In this process, the weights and thresholds need to be continuously modified. By adjusting the weight of each node in the network in real time, the input of the BP neural network can gradually approach the expected output of the network. If the error of the network is within the allowable area, the training is terminated when the network error meets the accuracy requirements of the algorithm or the number of training steps exceeds the maximum number of steps. The specific process of the BP learning algorithm is as follows:

(1) Initialization of the network: the weights and thresholds of the network are initialized by random numbers in (−1, 1) to determine the maximum learning step size and allowable error area.
(2) Read the preprocessed training samples and the expected output value of the network.
(3) Calculate the output value of each hidden layer unit (for the qth sample).
  (2) $$\begin{array}{c} O_{qj}=f\sum_{i=1}\left(v_{ij}I_{qi}-\lambda_{j}\right)\text{.} \end{array}$$
(4) Calculate the error signal of each layer node Output layer:
  (3) $$\begin{array}{c} \delta_{qk}=o_{qk}\left(y_{qk}-o_{qk}\right)\left(1-o_{qk}\right)\text{.} \end{array}$$
Hidden layer:
  (4) $$\begin{array}{c} o_{qi}=o_{qi}\left(1-o_{qi}\right)\sum_{i=1}\delta_{qi}v_{ij}\text{.} \end{array}$$
(5) Back propagation of error signal Weight correction:
  (5) $$\begin{array}{c} V_{ij}\left(t+1\right)=\partial \delta_{qi}o_{qi}+V_{ij}\left(t\right)\text{.} \end{array}$$
Threshold correction:
  (6) $$\begin{array}{c} \lambda_{j}\left(t+1\right)=\lambda_{j}\left(t\right)+b\delta_{qi}\text{.} \end{array}$$
(6) Calculate the global error
  (7) $$\begin{array}{c} E_{q}=\left(\sum_{q}\sum_{k}\right)\frac{{\left(o_{qk}-Y_{qk}\right)}^{2}}{2}\text{.} \end{array}$$
(7) If the network error is within the allowable area, when the network error meets the accuracy requirements of the algorithm or the number of training steps exceeds the maximum number of steps, the training is terminated. On the contrary, carry out a new round of learning.

To build a logistics demand forecasting model, it is necessary to understand the historical data of local freight volume and related factors. The basic principles of regional logistics demand forecasting are divided into two parts: first based on the gray GM (1, N) forecasting model, forecast the change range of freight volume in the region and obtain the model forecast result and forecast residual. The forecast results are used to roughly show the law of the range of freight volume changes in the region. Second, use the BP neural network model to correct the prediction residuals obtained in the first step to obtain the final prediction result of regional freight volume. The principle of forecasting regional logistics demand is shown in Figure 2.

The following original relevant forecast data come from the National Bureau of Statistics, and the data results are highly authoritative, as show in Table 1. Experimental raw data graph as show in Figure 3.

This paper uses the GM(1, 1) model to simulate Beijing's freight volume data from 2010 to 2015. The specific calculation results are as Table 2.

Different from the GM (1, 1) model, the GM (1, N) model is a multivariate forecasting model, so it is necessary to consider the role of related factors when estimating Beijing's logistics demand. In this model, Beijing's freight traffic data was selected as the system feature sequence from 2007 to 2015. The five predictive index data include the output value of the primary industry, the output value of the secondary industry, and the output value of the Beijing area from 2007 to 2015. The consumption level of Beijing residents, the size of the population and the fixed asset investment of the whole society serve as the sequence of related factors.  Table 3 shows the data after initialization.

As show in Figure 4, we can see that the average relative error of the GM (1,6) model is only 3.57%, which shows that the prediction accuracy of this model is high, and it can predict the range of changes in Beijing's freight volume.

## 4. Logistics Finance Collaborative Development Model

### 4.1. The Formation of Logistics Finance

The formation of the logistics financial model is inseparable from the close integration of the logistics industry and the financial industry, as well as the attention and strong support of logistics companies, financial companies and financing institutions. China's small- and medium-sized enterprises play a huge role in increasing employment, promoting growth and technological innovation, and are the most dynamic and critical component of China's economic structure. Since SMEs are mostly companies with light assets and low credit ratings, the traditional bank credit system is cautious in granting loans to SMEs, and financing problems have long restricted the development of SMEs. As the barriers to entry into the banking industry continue to decrease and competition in the financial market becomes fierce, banks and other financial institutions continue to expand their business channels in order to consolidate their positions. However, due to the difficulty of credit risk management and control for SMEs, they are still cautious in financing business. In China, the threshold for starting a logistics company is low, which has resulted in a large number of logistics companies in China, especially small logistics companies founded by individuals. Under the background of this low-level competition, China's domestic logistics companies have low overall profit margins. In order to deal with this situation, logistics companies have to develop new value-added logistics services to expand profit margins and further development.

So far, the basic model of logistics finance is mainly divided into three parts, including logistics settlement finance, logistics warehouse receipt finance, and logistics credit finance. Among them, the most important model with the largest proportion is logistics settlement finance, which refers to a financial method that provides loans to individual service objects, logistics companies, and financing companies through various convenient and efficient settlement methods. There are three major parts: payment collection business, advance payment business, and acceptance bill business.

Regarding financial logistics, it is indeed a new concept recently, and it is indeed a development trend in the future. Regarding “logistics finance,” in fact, the literal interpretation is still “finance” + “logistics,” but they were once two unrelated things that were combined to operate. To explain this, we have to start with corporate financing. When it comes to corporate financing, most people can think of are bank acceptance bills, and working capital loans. Although these are tools to solve the capital gap in the actual production of enterprises, they are still on the surface after all. In general, to support enterprise production, it is necessary to analyze the production links of the enterprise. There are three processes in the production process of an enterprise. To put it in a popular language, it is the three stages of purchasing raw materials-production-sales and payment collection. Without considering any collateral such as the company's land, workshops, a production is functioning normally. For the above three processes, there are three financing modes: prepaid account financing, spot financing, and accounts receivable financing.

In fact, it is not difficult to find at this time that these three financing modes are closely related to “goods.” In fact, they use goods that the company will purchase, goods that have been produced, and goods that have been sold but have not yet received payment. The goods are used as collateral for financing. The concept of “logistics finance” was put forward, first of all, banks have the need to manage goods, and second, major warehousing and logistics companies have experience in managing warehouses and willingness to make money, and finally developed our first trade finance and goods-related product, spot pledge. What is spot pledge? It means collateral financing for the goods that have been bought in the warehouse or the goods that are produced for sale. At this time, the right of the goods belongs to the credit enterprise itself. The bank issues loans and uses the logistics company to manage the warehouse to ensure the goods Safety. At the same time, it is necessary to solve the prepayment problem. The solution is simple. The bank helps the borrower buy the goods, and the logistics company supervises the transportation at the same time. This forms a new future cargo rights pledge model. The bank buys the goods and the goods are supervised by the company. Acting as an agent for customs declaration, delivery, transportation, and finally into the borrower's own warehouse, and transferred to the spot pledge mode. At this time, the prototype of financial logistics has appeared.

After that, we once again carried forward on the basis of future cargo rights pledge. Aiming at the actual situation of core enterprises and various powerful upstream and downstream enterprises, we researched and developed a thing called “confirmation warehouse”. In fact, it is complicated to think about, but simple to say. Once again use the management ability of the logistics company with its own warehouse, entrust them to keep the goods, introduce the buyer and the seller to sign an agreement with the bank at the same time, once the buyer does not pick up the goods, the seller must promise a refund or repurchase the batch of products. Financial logistics appeared in China less than ten years ago, but it has flourished and there is still much room for development in the future. Combining the network coverage advantages of major logistics companies and the financial innovation capabilities of major banks, a more comprehensive logistics financial model is bound to emerge in the future.

### 4.2. Connotation Analysis of Coordinated Development of Logistics Finance

Whether the logistics financial system can develop harmoniously depends on whether the various parts of the system can merge with each other spontaneously, divide the work, realize the coordination and synchronization of all parts, and realize the seamless connection of all links. Strictly speaking, the coordination of the logistics financial system should include two parts: the coordination within the system and the coordination between the system and the external environment, as shown in the figure. The internal coordination of the system refers to the process of each subject in the system, based on a certain operation mode, the goal of maximizing the overall benefits of the system, and forming a healthy and orderly development status quo. Resource complementation and information sharing objects Under internal driving forces (including risk control and demand win-win). The ultimate goal of the coordinated development of logistics finance is to be able to use financial companies to provide financial assistance to the vast number of small- and medium-sized enterprises, while reducing the risks that exist in the financing process. While developing financing business, logistics finance has also obtained huge interest margins. Logistics companies can fully comply with the regulatory requirements of financial institutions for internal transactions in the supply chain and obtain certain benefits from supervision and information consulting services. While monitoring, they can effectively expand the business scope of the company and effectively solve the problems in the development of small- and medium-sized enterprises. We will try our best to solve the problem of insufficient capital turnover and break the funding bottleneck of the entire supply chain. Generally speaking, the ultimate requirement of collaborative development within the system is to make full use of the functions of the main body of the system, fully share system internal information, and make full use of resources. Meaning map of coordinated development of logistics financial system as show in Figure 5.

### 4.3. Collaborative Development Model of Logistics Finance

The continuous integration of the logistics industry and the financial industry has promoted the rapid development of logistics finance. Synergy theory emphasizes that through the coordination of various subsystems, jointly promote the orderly and stable operation of the entire system. Synergy theory plays an important role in logistics financial risk management and healthy development. In the 1970s, the famous physicist Harken founded the theory of synergy. According to the synergy theory, although different systems have different attributes and characteristics, there are mutual influences and synergy between different systems in the entire environment. This theory mainly studies how to make use of the synergy of its own internal subsystems when an open system is in an unstable state to make the system automatically form a stable and orderly structure in the dimensions of time, space, and function. Synergy theory includes three main contents, namely synergy effect, self-organization principle, and servo principle.

Synergy theory is suitable for logistics finance. If the economy is compared to a diversified and open system, then under the interaction of relevant subjects of the economic system, synergy becomes important. In other words, coordination is an indispensable condition for healthy and sustainable economic development. If the system participants can actively cooperate and cooperate around the long-term goals of the system, then all the stakeholders in the system will be harmoniously linked together to give full play to the synergy of the system. If system participants disregard the overall development and only consider their own short-term interests, in order to protect their own interests from damage, they will not hesitate to create friction, breach of contract or even conflict with other participants, then the entire system will become chaotic and unable to exert the system's application Some role. Therefore, enterprises must reasonably coordinate the internal links of the system, determine the impact of the coordinated development of logistics and finance, and make up for their own shortcomings with the help of other corporate members in the system to promote the deep integration of the industry.

All parties should establish a coordination mechanism. The progress and development of logistics finance are inseparable from a complete and reasonable coordination mechanism. In addition, financial institutions should actively seek logistics companies with high credit, strong strength, and multiple customers to establish strategic partnerships, conduct cooperation between businesses, learn from the development experience of the logistics industry, and improve by sharing information Supply connections between customers and enterprises, clarify rights and responsibilities, improve restraint mechanisms, and provide financing services for financing enterprises. Financial institutions should try to avoid competition, strengthen cooperation, share the logistics information they collect, and avoid the risk of repeated pledge financing. Logistics companies also need information cooperation, especially the management of pledge supervisors. Only the close cooperation of the three parties can reduce the risks of logistics finance to the greatest extent. The establishment of a tripartite coordination and cooperation operating mechanism is the foundation for the healthy and sound development of logistics financial services in the future.

All parties should focus on long-term collaboration. To achieve long-term coordinated development, logistics companies, financial companies, and financing institutions must abandon the boundaries of pursuing short-term benefits, establish and consolidate long-term cooperative relationships, trust each other, and work together to research and develop more reasonable, more efficient and safer financial products, and finally realize common development and common progress. In addition to giving up the pursuit of short-term benefits, logistics companies, financial companies, and financing institutions need to cooperate and coordinate with each other. The government financial supervision department should give full play to its supervisory role, continuously revise, improve, and implement logistics financial business development norms, establish a unified national credit evaluation system and disciplinary system, strictly supervise all behaviors, and prevent illegal acts. For enterprises, establish a credit default blacklist system and a logistics financial risk early warning mechanism to create a safe, open and transparent market environment.

## 5. Conclusion

This paper develops a logistics financial system based on neural network, which can easily predict regional logistics demand. Finally, taking city B as an example, the system is used to analyze and forecast the cargo transportation volume of city B. By comparing and analyzing the prediction effects of the four prediction models in the system, it can be seen that the significant advantage of the neural network prediction algorithm is that it can accurately and reasonably predict the development needs of the logistics industry in city B in the next five years. Logistics finance is a brand-new financing model that can effectively integrate logistics enterprises, financial companies, and financing institutions to achieve mutual benefit and win-win results. It can be said that in the future competition, who can use logistics finance rationally and effectively will be able to take the lead in development. Logistics finance closely links small and medium-sized enterprises with banks and other financing departments. It not only solves the problem of corporate financing difficulties but also increases the proportion of logistics companies in the future market. The uncertainty of financial information, the motivation of each business service object to pursue high returns in a short period of time, the inadequate prerisk conditions, and the provision of false information by logistics companies have led to an unprecedented development of logistics financial services. Credit risk. The credit risk of logistics finance comes from information asymmetry and the short-sighted behavior of stakeholders. Therefore, it is necessary to establish a perfect mutual restraint, coordinated development restraint mechanism and a cross-industry information platform to promote the deepening of industrial integration.

## Figures and Tables

**Figure 1:** Cross-validation method diagram.

**Figure 2:** The principle of forecasting the scale of regional logistics demand.

**Figure 3:** Experimental raw data graph.

**Figure 4:** Fitting results of GM (1,6) model.

**Figure 5:** Meaning map of coordinated development of logistics financial system.

**Table 1:** Experimental raw data.

Years	*x*_1_	*x*_2_	*x*_3_	*x*_4_	*x*_5_	*x*_6_
2007	19877	101.26	2509.40	18553	1216.25	3907.20
2008	20525	112.83	2626.41	20113	1232.28	3814.73
2009	20470	118.29	2855.55	23023	1217.52	4616.92
2010	21762	121 36	3388.38	24982	1258.00	8102.95
2011	24663	136.27	3752.48	27760	1277.92	5578.93
2012	26162	150.20	4059.27	30350	1297.46	6112.40
2013	28748	159.64	4202.86	33337	1316.34	6847.06
2014	26551	158.99	4544.80	36057	1333.40	6924.23
2015	20078	140.21	4542.64	39200	1345.20	7195.99

**Table 2:** Fitting results of GM(1, 1) model.

Years	Actual value	Analog value	Residual	Similarity error
2010	21762	21762.00	—	—
2011	24663	20321.79	−1660.79	6.73%
2012	26162	25454.36	707.64	2.70%
2013	25748	21613.64	1134.36	4.41%
2014	26551	28600.70	2750.3	10.36%
2015	20078	23014.60	−2936.6	14.6%

**Table 3:** Data after initialization.

Years	*x*_1_	*x*_2_	*x*_3_	*x*_4_	*x*_5_	*x*_6_
2007	1	1	1	1	1	1
2008	1.033	1.114	1.047	1.084	1.013	0.976
2009	1.03	1.168	1.138	1.187	1.026	1.182
2010	1.095	1.228	1.35	1.347	1.034	1.383
2011	1.241	1.346	1.495	1.496	1.051	1.428
2012	1.316	1.483	1.618	1.636	1.067	1.546
2013	1.295	1.377	1.71	1.797	1.082	1.752
2014	1.336	1.57	1.811	1.943	1.096	1.772
2015	1.01	1.385	1.81	2.113	1.106	1.919

## Data Availability

The data used to support the findings of this study can be obtained from the corresponding author upon request.
